The article "A Prospective Comparison of Three Strategies for Evaluating Blood Loss in Transurethral Resection of the Prostate" was published in 2021. Journal: Biomed Res Int.

# A Prospective Comparison of Three Strategies for Evaluating Blood Loss in Transurethral Resection of the Prostate

**DOI:** 10.1155/2021/8875380

**Published:** 2021-04-07

**Authors:** Xiaojuan Yuan, Wei Yu, Ronghua Wu, Longkun Li, Fan He

**Affiliations:** The Department of Urology, Second Affiliated Hospital, Army Medical University, Chongqing 400037, China

## Abstract

**Objective:**

The aim of the current investigation is to develop a new strategy for evaluating blood loss in the process of transurethral resection of the prostate (TURP).

**Methods:**

318 patients diagnosed with benign prostatic hyperplasia (BPH) that need TURP were enrolled in this study. Hospitalization information including age, height, weight, surgery time, prostate volume, hemoglobin (Hb) concentration, hematocrit (HCT) percentage, and red blood cell count (RBC) was evaluated for each patient. All statistical analysis drawing were conducted using R software.

**Results:**

Three methods were employed for calculating blood loss in TURP. Results from a new method display 0 missing value and got higher confidence (0 of 318, Poisson distribution, *P* < 0.001) compared with blood loss calculated with hemoglobin concentration (20.44%) and hematocrit percentage (19.18%). Also, the new method demonstrated narrow range (0.03~270.03 ml) and approximate normal distribution compared with blood loss calculated with hemoglobin concentration and hematocrit percentage. More importantly, the new method explained positive correlation with prostate volume (*R*^2^ = 0.138, *P* < 0.001) and also surgery lasting time (*R*^2^ = 0.193, *P* < 0.001).

**Conclusion:**

Methods developed for calculating blood loss in TURP in the current study displayed more accurate and reasonable evaluation of bleeding, which can guide the transfusion blood for patients.

## 1. Introduction

Transurethral resection of the prostate (TURP) is the most common surgery for benign prostatic hyperplasia (BPH) [1]. Despite its minimally invasive operation, bleeding still shows a common morbidity within and after surgery [2]. Some severe bleeding even requires blood transfusion and influenced the hospitalization and hospital resources [3]. Although improvement of surgical skills, anesthesia, and pharmacologic agents can reduce bleeding rate, transfusion rates during TURP were reported to be as high as 20% and have no tendency to fall [4, 5]. Therefore, accurate and reasonable assessment of blood volume in the process of TURP is very important for patient's rehabilitation.

Rapidly and accurately evaluating blood loss during surgery, strictly controlling bleeding, and effectively measuring blood volume are an important part of the perfect operation and good at postoperative rehabilitation for patients [6]. There are no reliable method and literature report to judge the amount of blood loss in the process of TURP [7]. The main strategies to measure intraoperative blood loss in operating rooms are estimation based on the amount of blood absorbed by gauze and estimation based on the induced drainage. All of the above are estimated by observation, with large bias, errors, and low accuracy. In clinical lab, several methods have been referred for evaluating bleeding. Ekengren and Hahn [8], for the first time, used a HemoCue photometer analyzing low-concentration hemoglobin (Hb), which verified to be more accurate. Some scholars [9] used the urine-strip method to measure the intraoperative blood loss in 11 patients who underwent TURP, and the results indicate that the urine-strip and spectrophotometer method were found to be highly correlated. In 2010, Descazeaud et al. [10] used the ^51^Cr isotope labeling method to determine the amount of TURP bleeding. The ^51^Cr labeling method was used 1 day before and 3 days after the surgery. The results showed that the average RBC loss was 209 ml and the amount of bleeding was 507 ml. Univariate analyses showed that prostate volume, resected glandular tissue weight, preoperative RCV, and operative time were significantly associated with RBC loss. However, these methods endured costly, time-consuming character.

The article "A Prospective Comparison of Three Strategies for Evaluating Blood Loss in Transurethral Resection of the Prostate" was published in 2021. Journal: Biomed Res Int.

In the current investigation, our group develops a new method for evaluating bleeding in TURP and also compared with previous methods measured with hemoglobin concentration and hematocrit percentage. The new method demonstrated convenience and is fast and economic for clinical application.

## 2. Materials and Methods

### 2.1. Patients

318 patient diagnosed with BPH that need TURP in the Second Affiliated Hospital of Army Medical University during the period from June 2018 to April 2019 were enrolled in the current investigation. Patient inclusion criteria included (1) patients diagnosed with BPH and that need surgery according to the EAU guideline [11], (2) patients with normal coagulation function; and (3) patients with voluntary participation in the study and that signed informed consent. This study was conducted with the approval of the medical ethics committee of the Second Affiliated Hospital, Army Medical University. WHO dehydration assessment tool was employed to perform hydration status before and after surgery in the current investigation. The blood was taken before surgery anesthesia based on patients' consent. No presurgery infusion was done before blood collection. Hospitalization information including age, height, weight, surgery time, prostate volume, hemoglobin (Hb) concentration, hematocrit (HCT) percentage, and red blood cell count (RBC) was evaluated for each patient.

The article "A Prospective Comparison of Three Strategies for Evaluating Blood Loss in Transurethral Resection of the Prostate" was published in 2021. Journal: Biomed Res Int.

### 2.2. Blood Loss Measurement

In the current investigation, three methods for evaluating blood loss were compared with each other. Methods using hemoglobin concentration (formula (2)) and hematocrit percentage (formula (3)) were performed as previously described and widely used in clinical practice. A new strategy (formula (1)) for evaluating blood loss was reported firstly in the current study. Briefly, 2 ml blood was collected from each patient before TURP and was diluted in 3000 ml saline and the amount of red blood cell (cell/ml) was measured for standardization. In addition, within 2 hours after surgery, the amount of red blood cell was calculated in the saline flush. In addition, the amount of red blood cell was calculated by using routine urine analysis. According to the red blood cell measurement before and after surgery, we calculated the blood loss in the process of TURP by the following formula:

(1) $$\begin{array}{c} \text{Formula }1:\text{calculated blood loss }\left(\text{ml}\right)=\text{RB}{\text{C}}_{\text{after}}/{\text{RBC}}_{\text{before}}\times {\text{saline}}_{\text{after}}/3000\times 2, \end{array}$$

where RBC_before_ is preoperative red blood cell in saline (cell/*μ*l), RBC_after_ is postoperative red blood cell in saline (cell/*μ*l), and saline_after_ is total volume of flush saline after surgery.

(2) $$\begin{array}{c} \text{Formula }2:\text{calculated blood loss }\left(\text{ml}\right)=\left({\text{Hb}}_{\text{before}}-{\text{Hb}}_{\text{after}}\right)\times 40, \end{array}$$

where Hb_before_ is preoperative hemoglobin concentration (g/l), Hb_after_ is postoperative hemoglobin concentration (g/l), and 40 (ml) is a value assuming in normal adult (70 kg weight, 5000 ml volume blood, 12.5 g/l hemoglobin) hemoglobin loss 1 g/l equals 40 ml blood loss (see reference [12]).

(3) $$\begin{array}{c} \text{Formula }3:\text{calculated blood loss }\left(\text{ml}\right)=\left({\text{HCT}}_{\text{before}}-{\text{HCT}}_{\text{after}}\right)/{\text{HCT}}_{\text{before}}\times 0.07\times 1000, \end{array}$$

where HCT_before_ is preoperative hematocrit percentage (%) and HCT_after_ is postoperative hematocrit percentage (%) (see reference [13]).

### 2.3. Statistical Analysis

Clinical characteristics were demonstrated as range (min~max value) and mean ± SD (standard deviation). Poisson distribution was used for comparing rate. All statistical analysis drawings were conducted using R software (http://www.R-project.org/).

## 3. Results

### 3.1. Demographic Characters

318 male patients with BPH receiving TURP were enrolled in current research. All clinical characters are displayed in Table 1. Age range was from 48~92 years old; the average (mean) and standard deviation (SD) of BMI is 23.65 ± 3.49. In addition, the range of surgery lasting time shows from 10 to 85 minutes, and prostate volume is 20~79.8 ml. Pearson correlation was calculated among clinical characters (Figure 1). The results showed that age was negatively correlated with height, weight, hemoglobin concentration, and hematocrit percentage, which was consistent with the actual situation. More importantly, surgery lasting time, prostate volume, and blood loss volume (calculated with formula (1)) were found positively correlation with each other.

The article "A Prospective Comparison of Three Strategies for Evaluating Blood Loss in Transurethral Resection of the Prostate" was published in 2021. Journal: Biomed Res Int.

### 3.2. Three Strategies for Evaluating Blood Loss

Three methods were employed for calculating blood loss (see Materials and Methods). The results show that blood loss calculated with formula (1) demonstrated a narrow range from 0.03 to 270.03 ml compared with blood loss calculated with formula (2) (range, 0~2160 ml) and formula (3) (range, 0~2079 ml) (Figure 2(a)). In addition, blood loss volume calculated with hemoglobin concentration and hematocrit percentage has 20.44% (65 of 318) and 19.18% (61 of 318) of 0 value, which was higher than blood loss calculated with formula (1) (0 of 318, Poisson distribution, *P* < 0.001). Distribution of blood loss volume was drawn with histogram with density curve fitting, and the results dedicated that the method calculated with formula (1) got a narrow range and approximate normal distribution (Figure 2(b)) compared with skewed distribution of methods calculated with formula (2) (Figure 2(c)) and formula (3) (Figure 2(d)).

### 3.3. Correlation with Blood Loss, Prostate Volume, and Surgery Lasting Time

Except a more accurate evaluation of blood loss, the method calculated with formula (1) demonstrated positive correlation with prostate volume (Figure 3(a), *R*^2^ = 0.138, *P* < 0.001) and also surgery lasting time (Figure 3(b), *R*^2^ = 0.193, *P* < 0.001). Conversely, we did not find any correlation between blood loss volumes calculated with formula (2) or formula (3) with prostate volume and surgery lasting time (Figures 3(a) and 3(b)).

## 4. Discussion

Based on the important role of evaluating blood loss in the surgery of TURP, the current study describes a method using red cell count (RBC) in flush saline as a reference. Actually, the new method was more accurate for evaluating bleeding and specially displayed better in counting range, variance, fitting curve, and also correlation with prostate volume and surgery lasting time compared with traditional evaluating methods. The advantage of the current method showed in several ways.

The article "A Prospective Comparison of Three Strategies for Evaluating Blood Loss in Transurethral Resection of the Prostate" was published in 2021. Journal: Biomed Res Int.

In the process of evaluating blood loss, formula (2) and formula (3) get results lesser or equal to zero, and this is because postoperative hemoglobin concentration or hematocrit percentage was more or equal to preoperative hemoglobin concentration or hematocrit percentage. Blood loss volume calculated with hemoglobin concentration and hematocrit percentage has 20.44% (65 of 318) and 19.180% (61 of 318) of 0 value, but not in blood loss calculated with formula (1) (0 of 318, Poisson distribution, *P* < 0.001). Several reasons can explain this phenomenon. Firstly, a test error was present in clinical lab in the case of a small amount of bleeding [14]. Secondly, the most important reason for hemoglobin or hematocrit percentage rising after surgery was due to different operation lasting times and the patient's fasting time before surgery. In a patient with short surgery time, there is no or a small amount of infusion in TURP, and then, the formation of blood physiological concentration is present after surgery [15].

Among the above various methods mentioned in instruction for determining the amount of bleeding during TURP, HemoCue photometer method, urine-strip method, and pectrophotometer method and the ^51^Cr isotope labeling method have high accuracy, good repeatability, and simple operation and are worthy of clinical application. However, still, some limitation must be mentioned for the above three methods. Although urine-strip and pectrophotometer methods are low in cost, the reliability of the results needs to be improved mainly due to manual production, measurement, and analysis [9]. The principle of the urine-strip and pectrophotometer method is characterized by heme in Hb of RBC having the activity of peroxidase which can catalyze the release of new ecological oxygen by hydrogen peroxide [16]. However, this method will cause technical errors because of the skill problems of the observer during the dilution and interpretation process, resulting in the measured amount of bleeding being 0.5 to 2 times compared with the actual value. With the HemoCue photometer method, it is important to ensure that the RBC is completely hemolyzed in the blood-containing drain to release free Hb to improve accuracy. Calibration of the instrument is the key in the process [17]. Although the ^51^Cr isotope labeling method is the most accurate, there are deficiencies in costly, time-consuming, cumbersome instruments and specialized technicians. According to the existing research, there is currently no measurement method that is considered a gold standard [18]. With the development of science and technology and the interdisciplinary application of multiple disciplines, each measurement method will be continuously improved, providing an important research tool for further strengthening intraoperative management, guiding postoperative treatment, and evaluating various new surgical methods. Therefore, bleeding measurement with new developed methods shows accurate, feasible, and cost-effective results. This method for measuring the amount of bleeding in TURP may become an optical choice.

The article "A Prospective Comparison of Three Strategies for Evaluating Blood Loss in Transurethral Resection of the Prostate" was published in 2021. Journal: Biomed Res Int.

## 5. Conclusion

In conclusion, a new method developed for evaluating bleeding in TURP shows to be accurate, feasible, and cost-effective in clinical application which deserves to be widely used in clinical practice.

## Figures and Tables

**Figure 1:** Heat map plot of Pearson correlation between clinical characterizations including age, height, weight, BMI, prostate volume, and surgery_time and parameters for evaluating blood volume in the surgery of TURP including Hb_before (hemoglobin value before surgery), Hb_after (hemoglobin value after surgery), HCT_before (hematocrit percent before surgery), HCT_after (hematocrit percent after surgery), Hb_count (blood volume evaluation according to hemoglobin value), HCT_count (blood volume evaluation according to hematocrit percent), and Newmethod_count (blood volume evaluation according to formula in methods).

**Figure 2:** Blood loss evaluations with three different methods: (a) comparison of blood loss volume (boxplot for mean and variance) in the surgery of TURP with three methods; (b) histogram for blood volume and fitting a density curve with new methods in the process of evaluation blood; (c) histogram for blood volume and fitting a density curve with hemoglobin value in the process of blood evaluation; (d) histogram for blood volume and fitting a density curve with hematocrit value in the process of blood evaluation.

**Figure 3:** Plot relationships between prostate volume, surgery time, and blood volume with three different methods for evaluating.

**Table 1:** Clinical characteristic of 318 samples including in current evaluation.

	Range (min~max)	Mean ± SD
Age (year)	48~92	70.58 ± 8.51
Height (m)	1.37~1.8	1.62 ± 0.06
Weight (kg)	26~100.4	62.26 ± 10.4
BMI		23.65 ± 3.49
Surgery_time (min)	10~85	43.06 ± 19.32
Volume (ml)	20~79.8	40.76 ± 15.19
Hb_before (g/l)	66~171	130.63 ± 15.99
Hb_after (g/l)	63~166	124.91 ± 16.03
Hb_count (ml)	0~2160	269.18 ± 288.59
HCT_before (%)	16.1~52.1	39.45 ± 4.75
HCT_after (%)	11.9~50.9	37.7 ± 4.73
HCT_count (ml)	0~2079	219.64 ± 246.5
Newmethod_count (ml)	0.03~270.03	23.39 ± 32.38

## Data Availability

The corresponding data of this manuscript can be available if any researcher required.
